# Applying Game-Based Approaches for Physical Rehabilitation of Poststroke Patients: A Systematic Review

**DOI:** 10.1155/2021/9928509

**Published:** 2021-09-14

**Authors:** Soheila Saeedi, Marjan Ghazisaeedi, Sorayya Rezayi

**Affiliations:** Health Information Management Department, School of Allied Medical Sciences, Tehran University of Medical Sciences, Tehran, Iran

## Abstract

**Objective:**

A large number of patients need critical physical rehabilitation after the stroke. This study aimed to review and report the result of published studies, in which newly emerged games were employed for physical rehabilitating in poststroke patients.

**Materials and Methods:**

This systematic review study was performed based on the PRISMA method. A comprehensive search of PubMed, Scopus, IEEE Xplore Digital Library, and ISI Web of Science was conducted from January 1, 2014, to November 9, 2020, to identify related articles. Studies have been entered in this review based on inclusion and exclusion criteria, in which new games have been used for physical rehabilitation.

**Results:**

Of the 1326 retrieved studies, 60 of them met our inclusion criteria. Virtual reality-oriented games were the most popular type of physical rehabilitation approach for poststroke patients. “The Nintendo Wii Fit” game was used more than other games. The reviewed games were mostly operated to balance training and limb mobilization. Based on the evaluation results of the utilized games, only in three studies, applied games were not effective. In other studies, games had effective outcomes for target body members.

**Conclusions:**

The results indicate that modern games are efficient in poststroke patients' physical rehabilitation and can be used alongside conventional methods.

## 1. Introduction

Stroke is one of the diseases that can lead to disability and affect people's daily activities and lead to reduced performance [1]. According to the Global Burden of Diseases (GBD 2010), stroke is the second most common cause of death worldwide [2]. In 2010, the number of people with the first stroke was 16.9 million, and people who died of stroke was 5.9 million [2]. Disability-adjusted life years (DALYs) lost also was 102 million, and the number of stroke survivors was 33 million [2]. Ninety percent of stroke survivors have a disability in one of their functions [3]. Most people with poststroke disability experience changes in emotional function, limb movement, balance, and muscle strength, and there is a risk of falling for these patients in performing ordinary activities, all of which affect the quality of life of survivors [4]. The main treatment solution to reduce functional defects after stroke is rehabilitation [5]. Poststroke physical rehabilitation in common is a gradual process that can take months or even years, and these patients require multiple sessions of treatment.

However, patients may not be able to attend these treatment sessions for rehabilitation fully. Several factors may lead to limited access to these treatment sessions, including the following: difficulty accessing a physiotherapist by the patient, high cost of attending the treatment session, patient's age and disability, the long distance that the patient has to travel, or poor patient compliance [6]. One of the solutions that can be offered to overcome these problems is to do rehabilitation activities at home; for rehabilitation exercises to be effective at home, high-intensity methods focused on specific repetitions of the practice with the feedback of performance should be used [7]. Consequently, one of the innovative methods that can obviate the above problems is applying modern games; these games have been used in various fields, including education, public policy, and healthcare [8]. Furthermore, they can also be utilized as a support tool for rehabilitation activities and provide an enjoyable environment for patients and increase adherence to treatment sessions [9, 10].

As it turns out, various studies have been performed to determine the effectiveness of the mentioned games. A systematic review study by Primack et al. found that games improved 69% of psychological therapy outcomes, 46% of clinician skills outcomes, 42% of health education outcomes, and 37% of disease self-management outcomes [11]. Another study examined the games managed for rehabilitation in respiratory conditions and concluded these games were effective [12, 13]. The purpose of this study is reviewing, summarizing, and reporting studies in which modern games have been used for physical rehabilitation of poststroke patients and tries to answer the following questions:

1. Which type of games is the most used?
2. Which gamification approaches have been used to improve the performance of poststroke patients?
3. What was the most common type of physical rehabilitation in stroke survivors?
4. What are the evaluation results of games used in poststroke patients?

## 2. Research Methodology

This systematic review was conducted based on Preferred Reporting Items for Systematic Reviews and Meta-Analyzes (PRISMA) checklist to ensure inclusion of relevant studies [14].

### 2.1. Design

In this review, a systematic search of scientific databases including ISI Web of Science, PubMed, IEEE Xplore Digital Library, and Scopus was performed from January 1, 2014, to November 9, 2020. The comprehensive search strategy comprised a set of main keywords from PubMed Mesh terms and Emtree related to “game,” “rehabilitation,” and “poststroke” patients. The specific detail of main applied keywords for each database is presented in Table 1.

### 2.2. Inclusion and Exclusion Criteria for Study Selection

The extracted studies were included if they fulfilled the following criteria: (1) original articles and proceedings, (2) the focus of this review was on only physical rehabilitation innovative game-based solutions for poststroke physical disabilities, (3) one of the gamification techniques was employed for physical rehabilitation or disability treatment, (4) in this study, the result of using different games and outcomes of video games or immersive-oriented approaches on physical rehabilitation were reviewed, and (5) studies were limited to those published in the English language. Besides, the studies were excluded if they met the following criteria: (1) the title, abstract, or full text of the article that did not relate to video games, virtual, or mixed reality-based games, (2) studies which were review or meta-analysis, book chapters, letter, reports, and technical reports, (3) articles in which the result of applying games was not reported quantitatively, (4) articles about cognitive rehabilitation, and (4) non-English published ones.

### 2.3. Literature Refinement

In comprehensive and scientific databases searching, 833 studies were retrieved after duplicate removal. Some inclusion and exclusion criteria were set for the study selecting phase. In the first phase, two independent reviewers (SS and SR) specified the primary classification of included studies; then, they synthesized selected citations' critical features. MG validated the primarily determined classifications. All titles and abstracts of extracted studies were investigated and screened based on the research questions and unique aims to select relevant ones by two reviewers under MG's supervision. In the last phase, citations that met inclusion and exclusion criteria were selected to enter the full-text review phase. The full-texts of relevant studies were screened by SS and SR thoroughly. Key characteristics were entered into a spreadsheet in Excel for each study. Two authors (SR and SS) independently extracted the study characteristics based on the predefined classifications. For reaching an agreement, the information was examined again by two authors. The next reviewer (MG) evaluated and validated all of the obtained results. EndNote X9 was used for resource management, and all qualitative analyses were performed in SPSS v20. The main classifications of screened citations are shown in Figure 1.

## 3. Results

The flow of screening articles based on the PRISMA method is shown in Figure 2. Prior scientific searches assigned 833 citations after the duplicate removal phase. Next, 41 studies were eliminated due to their irrelevancy in the full-text screening phase. In the last screening step, 60 studies were included based on our main study objectives as eligible studies. Based on the predefined classification elements, a summary of the key results is described in Table 2.

### 3.1. Study Characteristics

The reviewed studies in this study were published in 53 journals and 7 international conferences. All the names of journals and conferences are listed in Table 3 based on their frequency. As it is clear, the “Archives of Physical Medicine and Rehabilitation,” “Clinical Rehabilitation,” “Games for Health Journal: Research, Development, and Clinical Applications,” and “Journal of Stroke and Cerebrovascular Diseases” have the first rank with 5 or 4 published studies among journals. The distribution of studies by year and country of publication is presented in Table 4. As it is conducted, the majority of citations were published in 2019. Accordingly, in different countries, innovative physical rehabilitation solutions were employed and Korea with 13 citations had the highest number of studies.

### 3.2. The Distribution of Literature by Main Gamification Types and Approaches

Based on analysis, virtual reality-oriented games and video games are the most popular physical rehabilitation types for poststroke patients. The distribution of reviewed literature based on the type of games is shown in Figure 3. Besides, it turns out “Microsoft Xbox 360 Kinect” and “the Nintendo Wii Fit” approaches have been the widest utilized game-based tools that have been extracted in studies (Figure 4).

The deployment platform for most of the studies included in this review (*n* = 28, 46.66%) was Nintendo and Microsoft Xbox 360 Kinect.

There are many games in the field of rehabilitation that researchers and therapists can use for rehabilitating patients. However, in this systematic review, most studies have used existing games in rehabilitation and do not develop games for the purpose of research that we can refer to the Nintendo Wii Fit, Microsoft Xbox 360 Kinect games, Peggle, IREX, and HTC Vive games.

### 3.3. Distribution of Studies Based on Type of Physical Rehabilitation

The critical types of physical rehabilitation therapies applied for poststroke patients based on different games were divided into several main categories. The most important types of rehabilitation are “Balance training,” “Mobilization of the limbs,” and “Muscular strengthening” (Figure 5).

### 3.4. Distribution of Studies Based on Type of Studies, Sample Size, and Session Detail

In the investigated studies, three types of intervention studies and their effectiveness have been utilized (Table 5). The sample size from minimum to maximum number is 5 people in 2 studies and 209 people in one study. The highest frequency for the selected sample size was 10 people, which is in 4 studies. The lowest age of the recruited subjects in studies was 24 years on average, and the highest mean of age was 72 years old. In most studies, the number of males included in the intervention was higher than females; in 4 studies, the exact number of genders was not reported.

The frequency of physical rehabilitation time (by unit time) is shown in Figure 6. In this study, the length of rehabilitation time is converted to hour to compare the treatment time in different studies. In studies, the minimum duration of treatment to provide rehabilitation is one hour; besides, 10, 9, and 12 hours is the highest frequency of treatment time in studies, which was intended in a total of 12 studies.

### 3.5. Distribution of Studies Based on Assessment Scores

According to the results of reviewed different studies, numerous indicators and tests have been applied to evaluate physical rehabilitation outcomes in poststroke patients. In other words, according to the type of rehabilitation treatment provided to patients, different indicators and metrics have been calculated to assess the condition of the rehabilitated organs of the body (before and after the intervention). For this reason, we were unable to compare the assessment scores calculated during the intervention. However, considering how many indicators and metrics in each study were affected by physical rehabilitation during the intervention treatment, we added a brief assessment from the authors' perspective. At the end of the intervention, if all indicators of functional or physical appraisal of patients are affected by game-based rehabilitation and a significant difference is seen, then we have labeled this rehabilitation approach “Effective.” If only one or two of the several evaluation metrics are not affected by game-based rehabilitation, then we label them “Partly effective.” Finally, if there is no significant difference in all evaluation measures before and after the intervention, we label them “No effective.” In the following, the distribution of the reviewed studies based on effectiveness is shown in Figure 7.

## 4. Discussion

This survey's main objective was to review the studies in which games were applied for improving the physical functions and rehabilitation of poststroke patients. According to results, emerging games possess the capacity and potential to rehabilitate physical aspects in poststroke patients; furthermore, these games can help patients improve their independence. According to surveys, virtual reality-based approaches and “the Nintendo Wii Fit” games were used more than other games. The most common use of games in poststroke survivors' rehabilitation was related to limb movement and balance training.

Due to the included studies' results, different indicators and scales have been calculated and statistically analyzed to evaluate and test game-based physical rehabilitation therapies for poststroke patients. These statistical analyses demonstrated the positive effect of innovative rehabilitation is provided in the form of games for these patients. Even in many studies, applied games in different environments (virtual reality, and video-based games) have led to a great improvement in patients' physical problems such as balance disorder, upper extremity spasticity, and limbs' immobility and muscular weakness [3, 5, 11, 74–77]. Researchers in these studies have concluded that they can incorporate these games into the treatment plan and physiotherapy of poststroke patients and use them as alternative therapies to traditional methods because, in these experimental studies, significant improvements in all outcome measures were found after the intervention [76, 78]. However, in infrequent articles, no significant differences can be observed in all assessment scales (baseline and post-intervention assessments in the experimental and control groups) to evaluate game-oriented physiotherapies' effectiveness. For this reason, in these studies, the researcher has concluded that the game chosen to rehabilitate poststroke patients cannot be a useful tool to alternate with the traditional physical rehabilitation methods, and applying them can destroy the patient's time and motivation.

The reason for the ineffectiveness of newly emerged games for motor rehabilitation of stroke patients can have different reasons as follows: insufficient session times and training duration to generate consistent improvements in all patients, the insufficient number of participants in the experimental studies (randomized trails would require at least 25 participants in each group) [38, 76], the high mean age of patients in both intervention and control groups (underlying disability of people due to their age), and excessive movement limitations of the patients recruited in the study [79, 80].

According to this study's results, the most popular type of game for physical rehabilitation of poststroke patients was virtual reality games. Virtual reality-based games allow patients to interact with a virtual environment while performing rehabilitation exercises and simulating real functions. These games increase patients' motivation to perform rehabilitation exercises and provide a pleasant environment for patients, which can lead to more repetition of rehabilitation exercises in these patients [77]. People get feedback while playing virtual reality games, and this factor encourages patients with disabilities to attend therapy sessions and use their remaining functional capacity to succeed in the game [81].

Results have shown that “the Nintendo Wii Fit” games are used more than other games to rehabilitate poststroke patients. Several factors can lead to the most use of this game. Among these factors, we can mention the price of these games, which are relatively inexpensive. These games are widely available to people, and studies have shown that providing an attractive environment increases patients' enjoyment and more repetition of rehabilitation exercises [82–84]. Features of the Wii Fit game system lead to the stimulation of people's interest in continuing to play and can be useful for improving motor function and balance control [61].

Studies showed that the most common use of games in the rehabilitation of stroke survivors was related to limb movement and balance training. In other words, the results of studies that were run to examine the effect of games on people after a stroke had shown these games were effective in improving the balance of people and strengthening the muscles of the limbs [85]. In a systematic review conducted by Corbetta, the effectiveness of virtual reality games has been investigated and concluded that managed games have the most significant impact on patient mobility [75]. According to the results of this survey and other studies that show the effect of the game on maintaining balance and movement, it is recommended to use these games in poststroke survivors.

This systematic review had several strengths and limitations. One of the strengths was the use of broad keywords to search in 4 crucial databases. Another strength of this survey was the inclusion of studies presented at conferences. The limitations were the exclusion of articles in non-English language and the time limit imposed on searching databases (from 2014 onwards). Another limitation of this review was the different scales used to measure people's performance, and this factor made it difficult to compare the results of different surveys.

## 5. Conclusion

Game-based approaches lead to patients being able to smoothly perform their rehabilitation movement techniques without going to the treatment centers. These games can immerse the person in the environment by providing virtual or augmented reality capabilities and multiplying the effectiveness of the treatment. Therefore, the use of appropriate technology-based gaming solutions can improve patients' treatment and minimize the waste of time and cost of providing traditional motor rehabilitation. Consequently, these game-based treatments are considered complementary to traditional ones and can reduce the workload of therapists and accelerate the rehabilitation process. Future research should focus on how task-specific game-oriented systems can improve function after stroke, and statistical studies can show this effect more.

## Figures and Tables

**Figure 1:** The key classification of relevant studies.

**Figure 2:** The PRISMA diagram for the records search and study selection.

**Figure 3:** The distribution of studies based on gamification types.

**Figure 4:** The distribution of studies based on type and name of games.

**Figure 5:** Physical rehabilitation therapies in reviewed studies.

**Figure 6:** The distribution of studies based on the total time of rehabilitation duration.

**Figure 7:** The distribution of the reviewed studies based on effectiveness.

**Table 1:** Search strategy for each database.

Database	Search strategy
PubMed	(“Stroke”[Mesh] OR “cerebrovascular accident” OR “cerebrovascular accidents” OR “CVA” OR “CVAs” OR “cerebrovascular apoplexy” OR “brain vascular accident” OR “brain vascular accidents” OR “cerebrovascular stroke” OR “cerebrovascular strokes” OR “apoplexy” OR “cerebral stroke” OR “cerebral strokes” OR “acute stroke” OR “acute strokes” OR “acute cerebrovascular accident” OR “acute cerebrovascular accidents”) AND (“video games”[Mesh] OR “game” OR “games” OR “gamification” OR “video game” OR “computer games” OR “computer game”) AND (“rehabilitation”[Mesh] OR “rehabilitation care”) limit to: 2014–2020
Scopus	TITLE-ABS-KEY (( “stroke” OR “cerebrovascular accident” OR “cerebrovascular accidents” OR “CVA” OR “CVAs” OR “cerebrovascular apoplexy” OR “brain vascular accident” OR “brain vascular accidents” OR “cerebrovascular stroke” OR “cerebrovascular strokes” OR “apoplexy” OR “cerebral stroke” OR “cerebral strokes” OR “acute stroke” OR “acute strokes” OR “acute cerebrovascular accident” OR “acute cerebrovascular accidents”) AND (“video games” OR “game” OR “games” OR “gamification” OR “video game” OR “computer games” OR “computer game”) AND (“rehabilitation” OR “rehabilitation care”)) AND (limit to (pubyear, 2014–2021)) AND (limit to (doctype, “cp”) OR limit to (doctype, “ar”) AND (limit to (language, “English”))
Web of Science	TS = (“Stroke” OR “cerebrovascular accident” OR “cerebrovascular accidents” OR “CVA” OR “CVAs” OR “cerebrovascular apoplexy” OR “brain vascular accident” OR “brain vascular accidents” OR “cerebrovascular stroke” OR “cerebrovascular strokes” OR “apoplexy” OR “cerebral stroke” OR “cerebral strokes” OR “acute stroke” OR “acute strokes” OR “acute cerebrovascular accident” OR “acute cerebrovascular accidents”) AND TS = (“video games” OR “game” OR “games” OR “gamification” OR “video game” OR “computer games” OR “computer game”) AND TS = (“rehabilitation” OR “rehabilitation care”)
	Refined by: document types: (article OR proceedings paper)
	Timespan: 2014–2020. Indexes: SCI-EXPANDED, SSCI, A&HCI, ESCI.
IEEE Library	((((((“All metadata” : “stroke”) OR “all metadata” : “cerebrovascular accident”) OR “all metadata” : “cerebral strokes”) AND “all metadata” : “game”) OR “all metadata” : “computer game”) AND “all metadata” : “rehabilitation”). Filters applied: 2014–2021

**Table 2:** Main characteristics of included studies.

No.	Authors	Year	Name of gamification approach	Type of gamification approach	Type of rehabilitation	Rehabilitated target members	Study design	Sample size	Sample description (sex, age (year))	Session details	Assessment time	Assessment score	Effectiveness	Results
1	Laffont I et al. [15]	2019	Not mentioned	Video game	Mobilization of the limbs	Shoulder, arm, and hand	RCT	51	AgeM = 58: male = 31 and female = 20	45 min, 5 sessions in a week for 6 weeks	Baseline and postintervention at the end of the program, between days 45 and 60 and follow-up at 6 months	In the subacute stroke stage, a difference of 9/10 points on the UL-FMS is considered, and BBT minimally detectable change is gained to be 5.5 blocks/min.	Effective	Post hoc analysis showed that scores in UL-FMS or BBT were significantly higher in the VG group than in the CR group
2	Cikajlo I et al. [16]	2020	Nintendo Wii Fit	Virtual reality game	Balance training	Legs	RCT	20	AgeM = 50.3: male = 15 and female = 2	15 min, 5 sessions for 1 week	Baseline and postintervention	Significant differences between the groups were found with the eyes closed, sharpened Romberg test (*p*=0.05), and standing on the right leg (*p*=0.035).	Effective	Video games enable independent balance training is feasible without strenuous physiotherapy.
3	Glueck AC and Han DY [17]	2019	Microsoft developed RoboRaid	Mixed reality game	Balance training	Legs	Before and after trial	14	AgeM = 25.21: male = 11 and female = 3	59.12 min, 35.71 days	Baseline and postintervention	MR game training provided significant reaction time improvements (*p* < 0.05) and vestibular performances (*p* < 0.05).	Effective	The results showed visuomotor reaction time, and balance metrics were significantly improved following MR game rehabilitation.
4	Ayoubi F et al. [18]	2020	Nintendo Wii Fit	Virtual reality game	Mobilization of the limbs	Shoulder, wrist, hand, and finger	Before and after trial	10	AgeM = 61.1: male = 5 and female = 5	30 min, 10 sessions, 2 days in 5 weeks	Baseline and postintervention	FMA scores revealed a significant improvement in the motor function (*p*=0.001). BBT scores increased from 12 pretherapy to 20.6 posttherapy, and the MAL-AOM scores increased from 1.09 pretherapy to 1.8 posttherapy.	Effective	Significant improvement in all outcome measures was found after the intervention.
5	de Gouvêa JX et al. [19]	2015	Nintendo Wii Fit	Virtual reality game	Mobilization of the limbs	Shoulder and elbow	Before and after trial	22	AgeM = 66.4: male = 15 and female = 7	60 min, 3 sessions in a week	Baseline and postintervention	Elbow flexion score (joint range of motion) increased from 127 to 134, and shoulder flexion score increased from 114 to 134.	Effective	Metrics showed that there were statistically significant improvements for all trained measures.
6	Cano-Mañas MJ et al. [20].	2020	Microsoft Xbox 360 Kinect	Video game with Kinect	Balance training Postural control Functionality	Not mentioned	RCT	48	AgeM = 63.13: male = 23 and female = 25	20 min, 24 sessions in 8 weeks.	Baseline and postintervention assessments: 8 weeks after the intervention	Significant differences resulted in the baropodometric (*p* < 0.01), the modified Rankin scores (*p* < 0.01), and the variable related to strength and the pain/discomfort dimension (*p* < 0.01) of the EQ-5D.	Effective	The findings show that applying a video game approach combined with conventional therapy may produce postural control, improvements in balance, functionality, and quality of life.
7	Şimşek TT and Çekok [21]	2015	Nintendo Wii Fit	Virtual reality game	Balance training Mobilization of the limbs	Shouler, wrist, and elbow	RCT	42	AgeM = 58.04: male = 29 and female = 13	45–60 min, 10 week, 3 days/week.	Baseline and postintervention assessment: after 10 weeks, after intervention, and treatment satisfaction after 10 sessions	A statistically significant difference was found between before and after treatment FIM (functional independence measure) scores (*p* < 0.05).	Partly effective	These results indicated the Nintendo Wii Fit training was as effective on daily living functions and quality of life in subacute stroke patients.
8	Hung JW et al. [22]	2019	Kinect2Scratch	Video game with Kinect	Mobilization of the upper limbs	Shoulder, elbow, and forearm	RCT	33	AgeM = 58.98: male = 22 and female = 11	30 min, 24 sessions in 12 weeks	Baseline, postintervention, and at the 3-month follow-up.	The total activity scores of the training on upper extremity was significantly higher in the Kinect2Scratch group than in the therapist-based training group (*p* < 0.001)	Effective	The application of Kinect2Scratch-oriented games may indicate a complementary strategy to conventional therapy for decreasing the therapists' workload.
9	Adie K et al. [23]	2016	Nintendo Wii Fit	Virtual reality game	Mobilization of the arms	Arm	RCT	209	AgeM = 67.3: male = 105 and female = 104	45 min, 42 sessions in 6 weeks	Baseline and postintervention after 6 weeks and six months	There was no significant difference in the primary outcome of affected arm function at six weeks follow-up (*p*=0.12) and no significant difference in secondary outcomes.	No effective	The results indicated that the Wii^TM^ was not superior to arm exercises in home-based rehabilitation for stroke survivors with arm weakness.
10	Ahmad MA et al. [24]	2019	Not mentioned	Virtual reality game	Mobilization of the upper limbs	Not mentioned	Before and after trial	34	AgeM = 63: male = 31 and female = 5	30 min, 8 sessions in 8 weeks	Baseline and postintervention on completion of the 8 weeks	The results showed a significant time-group interaction effect for IMI (*p*=0.001), Lawton IADL (*p* = 0.01), and SIS domain of communication (*p*=0.03). A significant time was found in FMA-UE (*p*=0.001), WMFT (*p*=0.001), and Lawton IADL (*p*=0.01).	Effective	The integration of VR games as an adjunct to standard physiotherapy for upper limb stroke rehabilitation was considered to be equally beneficial compared to standard physiotherapy.
11	Choi YH et al. [25]	2016	MoU-Rehab	Virtual reality game	Mobilization of the upper limbs	Shoulder, elbow, and wrist	RCT	24	AgeM = 66.55: male = 17 and female = 14	30 min, 10 sessions in 2 weeks	Baseline and postintervention on end of treatment and at 1 month	FMA-UE in experimental and control groups was calculated 34/67 and 53.75. Changes in the B-stage in exp and con groups were indicated 3.17–4.24 for the arm and 3.08–4.58 for the hand.	Effective	A larger improvement in the FMA-UE, B-stage, and MMT was found after treatment with the MoU-Rehab than with conventional therapy
12	Choi HS et al. [26]	2017	Nintendo Wii Fit	Virtual reality game	Balance training Lower extremity	Not mentioned	RCT	36	AgeM = 61.91: male = 21 and female = 15	30 min, 12 sessions in 4 weeks	Baseline and postintervention	Post hoc analysis revealed significant differences in AP-axis, and sway area; weightbearing symmetry of the game-based CIMT group is compared with the other groups (*p* < 0.05).	Effective	Game-based CIMT was more effective at improving static balance control (AP-axis and sway area) and weightbearing symmetry compared with the other groups.
13	Choi HS et al. [27]	2019	Not mentioned	Virtual reality game	Mobilization of the upper limbs	Elbows, hands, wrists, and finger	RCT	36	AgeM = 58.97: male = 23 and female = 13	30 min, 15 sessions in 5 weeks	Baseline and postintervention assessment on end of 5 weeks	The difference between the GR mirror therapy group versus the conventional mirror therapy and control groups was statistically significant (*p* < 0.05).	Effective	It indicated that GR device-based mirror therapy is an intervention that improves upper extremity function, neck discomfort, and quality of life
14	de Paula Oliveira T et al. [28]	2015	Nintendo Wii Fit	Virtual reality game	Balance training	Not mentioned	RCT	23	AgeM = 50.21: male = 13 and female = 10	30 min, 14 sessions in 7 weeks	Baseline and postintervention assessment on 1-week AT and at a 2-month FU	The analyses of the FMA-LE score at FU for the control and experiment group are 21.39–24.58. The analyses of the BESTest score at FU for the control and experiment group are 75–83.	Effective	Balance training performed in virtual reality by using NWF was more efficient than conventional balance training
15	Givon N et al. [29]	2015	Nintendo Wii Fit	Virtual reality game	Balance training Mobilization of the upper limbs	Not mentioned	RCT	47	AgeM = 56.35: male = 28 and female = 19	60 min, 2 sessions in a week for 3 months	Baseline and postintervention, a 3-month intervention and at 3-month follow-up	Significant improvements were presented in both groups for gait speed (*F* = 3.9, *p*=0.02), grip strength of the weaker (*F* = 6.67, *p*=0.002), and stronger hands (*F* = 7.5, *p*=0.001). Daily steps and functional ability of the weaker hand did not increase in either group	Partly effective	Video and VR games can promote measures of physical activity of patients with chronic stroke.
16	House G et al. [30]	2016	The BrightArm^TM^	Virtual reality game	Mobilization of the upper limbs	Arm, hand, shoulder, and wrist	Before and after trial	7	AgeM = 69.7: male = 5 and female = 2	45–50 min, 16 sessions in 8 weeks	Baseline and postintervention, on each booster period, each consisting of 4 sessions over 2 weeks in 8 weeks	Range of motion improved for 18 out of 23 upper extremity movement variables (*p*=0.01) between pretournament and posttournament assessments.	Effective	The results indicate that BrightArm is effective in improving the range of motion of the upper extremity
17	Hsieh HC [31]	2018	Not mentioned	Video game	Walking Balance training	Not mentioned	RCT	56	AgeM = 58.5: male = 33 and female = 23	30 min, 3.5 hours/week, 10 weeks	Baseline and postintervention	The calculated metrics showed that the patients in the intervention group showed significantly better 10MWT (*p*=0.033), the CoPAP sway (*p*=0.01), and the sway area (*p*=0.006) than in the control group.	Effective	This game improves exercise compliance and promotes recovery of balance and mobility after stroke.
18	Hsieh HC [32]	2018	Not mentioned	Video game	Balance training	Leg	RCT	54	AgeM = 64.07	40 min, 3 sessions in 1 week for 12 weeks	Baseline and postintervention	Significant changes in CoP sway kinematics were observed in sway path (*p*=0.001), sway area (, *p*=0.002), and sway velocity (*p*=0.007). Balanced tests are the BBS test: *p*=0.001 and TUG test: *p*=0.001), and there was no significant change in the FABS test	Partly effective	This innovative gaming approach with adaptive PC games will be a useful therapy for stroke rehabilitation
19	Huang LL and Chen MH [33]	2016	Gardening digital game	Video game with Kinect	Mobilization of the upper limbs	Not mentioned	Before and after trial	10	AgeM = 61.20: male = 5 and female = 5	24 sessions in three sessions per week	Baseline and postintervention	Fugl–Meyer Assessment of motor function (increases of 9.30); the Box and Block Test of manual dexterity (increases of 5.80); higher functional independence measure (increases of 6.50); and range of motion measurement of the upper extremity proxima (increases of 5.56) and distal (increases of 3.83)	Effective	The gardening digital game is benefit to improve upper extremity motor function.
20	Khan RU et al. [34]	2019	Not mentioned	Video game	Muscular strengthening	Fist, wrist, and forearm	Before and after trial	5	AgeM = 24: male = 3 and female = 2	Not mentioned	Baseline and postintervention	The scores of 3 players were improved up to 150, 171, and 172, respectively, for 2 players, and there is not mainly improvement.	Partly effective	This result shows that an attractive environment and real-time feedback mechanism can improve the rehabilitation process.
21	Afsar SI et al. [35]	2018	Microsoft Xbox 360 Kinect	Virtual reality game	Mobilization of the upper limbs	Shoulder and elbow	RCT	35	AgeM = 66.43: male = 20 and female = 15	30 min, per day for 4 weeks	Baseline and postintervention	For the experimental group, the change of BBT (pre-to-postdifference) scores showed a significant improvement when compared to the control group (*p*=0.007), but the change of FMA-UE and the FIM scores for the experimental group were not significantly higher (*p*=0.057, *p*=0.677)	Partly effective	The Kinect-based game system in addition to conventional therapy has supplemental effectiveness for stroke patients.
22	Lee MM et al. [36]	2016	Canoe game	Virtual reality game	Trunk postural stability Balance training	Trunk muscles and leg	RCT	10	AgeM = 65.7: male = 5 and female = 5	30 min a day, 3 sessions a week for 4 weeks	Baseline and postintervention	Improvements in trunk postural stability, balance, and upper limb motor function were observed in the EG and CG, but were greater in the EG. The mean SUS scores in the EG and TG were 71 ± 5.2 and 74.2 ± 4.8, respectively.	Effective	Canoe game-based virtual reality training is a beneficial intervention for improving trunk postural stability, balance training, and upper limb motor in stroke patients.
23	Lee D and Bae Y [37]	2019	DBIVG	Video game	Trunk postural stability Walking	Trunk and leg	RCT	21	AgeM = 55.1: male = 14 and female = 7	30 min, 12 sessions in 4 weeks	Baseline and postintervention	The scores of TISssb, TISdsb, and TISco for the intervention group improved up to 5.9, 6.18, and 3.0. The score of DGI is calculated up to 17.27. The scores of TWT and TUGT decreased up to 42.27 and 39.32.	Effective	The analysis demonstrated DBIVG can improve trunk control and gait ability in patients with chronic stroke.
24	Lee SH et al. [38]	2019	HTC Vive	Virtual reality game	Mobilization of the upper limbs	Hand, shoulder, fingers, and wrist	Before and after trial	12	AgeM = 40.2: male = 7 and female = 5	30 min, 10 sessions 2-3 times a week	Baseline and postintervention	In five participants, scores showed improvement both in ARAT and BBT. ARAT (pretraining 22.3 and posttraining 31.1), BBT (pretraining 11.2 and posttraining 19.6), and MBI (pretraining 90.4 and posttraining 93.0)	Partly effective	This study indicates a fully immersive VR rehabilitation program can be used for upper extremity rehabilitation in patients with chronic stroke
25	McNulty PA et al. [39]	2015	Nintendo Wii Fit	Virtual reality game	Mobilization of the upper limbs	Shoulder, elbow, and wrist	RCT	41	AgeM = 58: male = 31 and female = 10	60 min, 10 consecutive weekdays	Prebaseline (14 days pretherapy), baseline, postintervention, and postintervention after six-month follow-up	The Wolf Motor Function Test (WMFT-tt) improved from 21 to 17 after Wii-based movement therapy, and Motor Activity Log Quality of Movement Scale scores improved from 67.7 to 102.4 after Wii-based movement therapy.	Effective	This result indicated Wii-based movement therapy is an effective upper limb rehabilitation poststroke
26	Nijenhuis SM et al. [40]	2016	MyoCI	Video game	Muscular strengthening	Arm and hand	RCT	19	AgeM = 60: male = 10, and female = 9	30 min, 6 sessions in a week for six weeks	Prebaseline (one week before training), baseline, and 1 week after training (postintervention) and two months after the end of training follow-up	The control group reported a higher training duration (189 versus 118 minutes per week). No differences in clinical outcomes over training between groups were found (*p* > 0.165).	No effective	An extra advantage of this arm and hand training over the conventional arm and hand exercises at home was not proven.
27	Paquin K et al. [41]	2015	Nintendo Wii Fit	Virtual reality game	Mobilization of the upper limbs	Hand, finger, and wrist	Before and after trial	10	AgeM = 72.1: male = 10	15 min, 16 sessions, 2 sessions per week, for 8 weeks	Baseline and postintervention	Significant improvements were resulted with the JHFT, BBT, and NHPT from pretesting to posttesting (*p*=0.03, *p*=0.03, and *p*=0.01, respectively). An increase in QOL from pretesting to posttesting is determined by the SIS (*p*=0.009).	Effective	Findings demonstrated important improvements occurred between pretesting and posttesting on 4 metrics.
28	da Fonseca EP et al. [42]	2016	Nintendo Wii Fit	Virtual reality game	Balance training	Legs, arms, trunk, and hip	RCT	27	AgeM = 52.4: male = 9 and female = 18	45 min, 20 sessions in 3 months	Baseline and postintervention	The number of falls was statistically significant (*p*=0.049) only in the treatment group. The differences in gait balance in the control group (*p*=0.047) is resulted.	Partly effective	The rehabilitation of gait balance in poststroke people applying virtual reality had the reduction of falls.
29	Rand D et al. [43]	2016	Microsoft Xbox 360 Kinect	Virtual reality game	Balance training Mobilization of the upper limbs	Legs, shoulder, elbow, and finger	RCT	24	AgeM = 62: male = 15 and female = 9	60 min a day, 6 times/week for 5 weeks	Baseline (an average of two assessments) and postintervention, and at the 4-week follow-up	ARAT extremely improved by 13.9% and 9.6% following the video games and traditional self-training programs. The scores for the Box and Block Test were 20.6 and 21.3 for pre and posttreatment in the experimental group.	Effective	Video games or self-training programs can be applied for practice repetitive upper extremity movements without the supervision of a clinician.
30	Shin JH et al. [44]	2015	RehabMaster™	Virtual reality game	Mobilization of the upper limbs	Upper limb and trunk	RCT	32	AgeM = 53.95: male = 24 and female = 8	30 min for 5 days per week for 4 weeks	Baseline and postintervention	The scores of FMA-UE, physical functioning were improved for pre and post treatment (experimental group) 35.5 up to 38.5 and 15 up to 20. Both groups exhibited significantly improved upper extremity function (*p*=0.001)	Effective	Results indicate that game-based VR rehabilitation has specific effects on health-related quality of life and upper extremity function
31	Shin JH et al. [45]	2016	The RAPAEL Smart Glove™	Virtual reality game	Mobilization of the upper limbs	Forearm, wrist, finger, shoulder, and elbow	RCT	46	AgeM = 58.5: male = 36 and female = 10	30 min, 20 sessions for 4 weeks	Baseline and postintervention in the middle of the treatment immediately after the intervention and 1 month after the intervention	The improvements in the game group were supported by significant FM-total: *F* = 6.48, *p*=0.006; FM-prox: *F* = 5.73, *p*=0.007; FM-dist: *F* = 4.64, *p*=0.024). The improvements in the JTTtotal in the game group was supported by significant JTTtotal: *F* = 4.073, *p*=0.032)	Effective	The game system used in VR-based rehabilitation might be an ideal rehabilitation tool for the distal upper extremity in stroke survivors.
32	Standen PJ et al. [46]	2016	Nintendo Wii Fit	Virtual reality game	Mobilization of the upper limbs	Arm, hand, shoulder, and finger	RCT	27	AgeM = 61: male = 16 and female = 11	20 min, 3 times a day, for 8 weeks	Baseline and postintervention four weeks (midpoint) and eight weeks (final)	There was a significantly greater change from baseline in the intervention group on midpoint wolf MFT strength (intervention group: 2.47; control group: 2.19), and two subscales of the final Motor Activity Log are improved (intervention group:12.80; control group: 12.53)	Effective	There is a greater improvement from baseline in the intervention group, so it is effective to use and help clinicians.
33	Rand D et al. [47]	2015	Microsoft Xbox 360 Kinect	Virtual reality game	Balance training Mobilization of the upper limbs	Not mentioned	RCT	12	AgeM = 63: male = 7 and female = 5	60 min, 5 times a week for 5 weeks	Prebaseline, baseline, postintervention, and 4 weeks after the intervention.	The scores of ARAT for the experimental game-based group improved from 30 up to 40, also the Box and Block Test improved for this group from 25 up to 30, and standing balance improved too from 16 *p* to 29.	Effective	These video games encouraged upper extremity movements and have potential to promote standing balance.
34	Kottink AIR et al. [48]	2014	Not mentioned	Virtual reality game	Mobilization of the limbs	Arm and hand	RCT	18	AgeM = 61.4: male = 13 and female = 5	30 min, 3 sessions in a week for 6 weeks	Baseline and postintervention	ARA and FM improvements were significant within both groups (*p* ≤ 0.009 for the main effect for session), with effect sizes (partial eta squared) of 0.47 and 0.53 for the ARA test and FM assessment, respectively.	Effective	The present study showed that both the arm and hand function improved after training.
35	Rand D et al. [49]	2014	Microsoft Xbox 360 Kinect	Video game	Mobilization of the limbs	Upper extremity	RCT	29	AgeM = 59: male = 17 and female = 12	60 min, 2 sessions per week for 3 months	Postintervention during the last month of the intervention and 1-2 weeks following the sessions	Participants in the VGG performed a median (IQR) of 271 (157–490) active purposeful movements compared to 48 (3–123) active purposeful movements in the TG (*z* = .3.0, *p*=0.001).	Partly effective	Video games elicited more UE purposeful repetitions and higher acceleration of movement compared with traditional therapy.
36	Jordan K et al. [50]	2014	Not mentioned	Virtual reality game	Mobilization of the limbs	Upper limb	Before and after trial	12	AgeM = 68.6	45 min, 3 sessions per week for 4–6 weeks	Baseline (t1), 4 weeks later (t2), within 1 week of completing the intervention (t3), and a final assessment was given 4 weeks later (t4).	No change in the FMA-UL scores between t1 and t2, indicating a stable baseline; a significant increase in the FMA-UL scores between t2 and t3; a significant increase in the FMA-UL scores between t2 and t4; and no change in the FMA-UL scores between t3 and t4	Effective	The intervention improved the arm function in survivors of chronic stroke.
37	Fan SC et al. [51]	2014	Nintendo Wii Fit	Virtual reality game	Mobilization of the limbs	Upper arm	RCT	20	AgeM = 64.4: male = 14 and female = 6	60 min, 3 sessions per week for 3 weeks	Baseline and postintervention (week 0), immediately after treatment (week 4) and four weeks after treatment (week 8).	Dunn's pairwise comparison showed that TTP contractions in the Wii group improved significantly more than that of the no-treatment group (*p* < 0.005).	Effective	In this pilot study, OTSVR gaming had immediate effects on motor recovery and provided motivation for treatment compliance in stroke patients.
38	McEwen D et al. [52]	2014	IREX	Virtual reality game	Mobilization of the limbs Balance training	Lower extremity	RCT	59	AgeM = 64.1: male = 32 and female = 27	30 min, daily sessions for 3 weeks	Before, immediately after, and 1 month after training	More individuals in the treatment group than in the control group showed reduced impairment in the lower extremity as measured by the Chedoke McMaster Leg Domain (*p*=0.04) immediately after training.	Effective	VR exercise intervention for inpatient stroke rehabilitation improved mobility-related outcomes.
39	Hung JW et al. [53]	2014	Nintendo Wii Fit	Video game	Balance training	Leg	RCT	28	AgeM = 54.4: male = 18 and female = 10	30 min, 2 sessions per week for 12 weeks	Baseline, postintervention, and at 3-month follow-up	At 3-month follow-up, the improvement in TUG and FR tests was maintained (time effect in TUG, *p*=0.03, partial ŋ 2 = 0.17; FR *p*=0.01, and partial ŋ2 = 0.22), but there was an increased fear of falling in both groups	Partly effective	Exergaming is enjoyable and effective for patients with chronic stroke.
40	Norouzi-Gheidari N et al. [54]	2019	Jintronix system	Virtual reality game with Kinect	Mobilization of the limbs	Upper extremity	RCT	18	AgeM = 49.9: male = 10 and female = 8	44 min, 2-3 sessions per week for 4 weeks	Baseline, postintervention, and 4-week follow-up	MAL-QOM and both mobility and physical domains of the SIS with mean difference of 1.0%, 5.5%, and 6.7% between the intervention and control groups, respectively) at postintervention.	Partly effective	Using virtual reality exergaming technology may be beneficial to upper extremity functional recovery.
41	Aşkın A et al. [55]	2018	KineLabs	Virtual reality game with Kinect	Mobilization of the limbs	Upper extremity	RCT	38	AgeM = 55.0: male = 27 and female = 11	60 min, 5 sessions per week for 4 weeks	Baseline and postintervention	Differences from baseline of FMA, MI, and AROM (except adduction of the shoulder and extension of the elbow) were greater in group A (*p* < 0.05).	Partly effective	Kinect-based VR training may contribute to the improvement of the UE motor function and AROM in chronic stroke patients.
42	Miranda CS et al. [56]	2019	Nintendo Wii Fit	Virtual reality game	Balance training	Lower limbs	RCT	29	AgeM = 50.96: male = 15 and female = 14	3 sessions for 1 week. Session 1: 60 min; sessions 2 and 3: 30 min	Baseline and postintervention, 1S (first session), 2S (2 days after the 1 session), and 3S (7 days after the 1 session) of training.	The analyses showed only a significant effect for the side (ANOVA : *F* = 27.80, *p* < 0.001, ES = 0.99).	Partly effective	People showed performance improvement after training with VR, but there was no transfer of the gains obtained to an untrained task with similar balance demands.
43	Fernandes AB et al. [57]	2014	“Paddle Panic Mini Game”	Virtual reality game with Kinect	Mobilization of the limbs	Upper extremity	Nonrandomized clinical trials	40	AgeM = 50.75: male = 20 and female = 20	Not mentioned	Baseline and postintervention	Comparing the participants' performance by ANOVA, there was a significant difference in the number of hits between the patients and healthy individuals' groups, according to the trials (*p*=0.008).	Effective	Patients with right brain injury responded better to the virtual reality game.
44	Morone G et al. [58]	2014	Nintendo Wii Fit	Video game	Balance training Standing Transferring Facilitation of movements	Paretic side, upper limb, and leg	RCT	50	AgeM = 60.16	20 min, 3 sessions per week for 4 weeks	Baseline and postintervention (third evaluation occurred one month after the end of rehabilitation)	Wii fit training was more effective than usual balance therapy in improving balance (BBS: 53 versus 48, *p*=0.004) and independency in activity of daily living (BI: 98 versus 93, *p*=0.021).	Effective	Balance training with game was found to be more effective than conventional therapy alone in improving balance and reducing disability in patients with subacute stroke.
45	Noveletto F et al. [59]	2020	MimPong	Video game	Muscular strengthening	Lower limb	Before and after trial	11	AgeM = 59.0: male = 6 and female = 5	12 min, 2 sessions per week for 10 weeks	Baseline and postintervention (three alternate days at the end of the program)	Significant effect sizes (*d*) were found for QFG strength (*d* = 0.5; *p*=0.021), QFG control (*d* = 1.1; *p* < 0.001), HSG strength (*d* = 1.1; *p*=0.001), HSG control (*d* = 1.5; *p*=0.003), functional mobility (*d* = 0.3; *p* < 0.001), gait speed (*d* = 0.4; *p*=0.007), and motor recovery (*d* = 1.0; *p* < 0.001).	Effective	Results indicate that the intervention of a SG with both the proper apparatus and evaluation system may effectively promote lower limb motor rehabilitation of hemiparetic stroke patients.
46	Junior VA dos S et al. [60]	2019	Nintendo Wii Fit	Virtual reality game	Mobilization of the limbs Balance training Sensory function improvement	Upper limb and lower limb	RCT	40	AgeM = 55.6: male = 23 and female = 17	50 min, 2 sessions per week for 2 months	Baseline and postintervention (second assessment after 2 months of treatment)	An improvement in the mean scores was observed after treatment independent of the allocation group with significant intragroup changes: 14.5, 10.5, and 10.4 for PNF, VR, and PNF/VR, respectively.	Partly effective	The use of a program combining virtual rehabilitation and PNF presented results that were comparable with those obtained with the isolated techniques.
47	Choi D et al. [61]	2018	Nintendo Wii Fit	Virtual reality game	Balance training Walking	Lower limb	RCT	28	AgeM = 50.25: male = 17 and female = 11	30 min, 3 sessions per week for 6 weeks	Prebaseline, baseline, and postintervention (1 week before and after training)	WVRT group showed significant improvements of +3.00 (5.25) in the BBS score and −1.92 (6.33) *s* in the TUG test, with all results being significantly better than those of the GBT group (*p* < 0.05).	Effective	The WVRT was a useful program for improving visual perception and postural balance in individuals with chronic stroke.
48	Borstad AL et al. [62]	2018	Recovery rapids	Virtual reality game with Kinect	Mobilization of the limbs	Upper limb	Before and after trial	16	AgeM = 49: male = 10 and female = 6	3 hours per day for 10 days over 2 weeks	Baseline and postintervention	The mean, median, and interquartile range for within-subjects change on the WMFT (rate/60 seconds) and MAL-QOM (0–5 scale) were 5.8 (3.7), 5.8, 2.7–9.4 and 0.74 (0.66), 0.46, 0.28–1.11, respectively.	Partly effective	Favorable changes in performance speed and quality of arm use were found in this study.
49	Noveletto F et al. [63]	2018	MyBalance	Video game	Balance training	Not mentioned	Before and after trial	18	AgeM = 55.3: male = 8 and female = 10	12 minutes per day in the first ten sessions and 20 minutes per day in the remaining sessions; 2 sessions per week for 10 weeks	Baseline and postintervention	Evaluated outcomes were better for all EG participants. The BBS test showed a balance improvement of 12.1 ± 7.8% with a large ES (0.9). The functional mobility assessed by the TUG test showed an improvement of 15.1 ± 7.4%, but ES was small (0.4).	Effective	The results of this study support the clinical potential of a biomedical SG for balance rehabilitation of hemiparetic stroke patients.
50	Carregosa AA et al. [64]	2018	Nintendo Wii Fit	Virtual reality game	Mobilization of the limbs Muscular strengthening Balance training Coordination	Upper limb and lower limb	Before and after trial	5	AgeM = 54.8: male = 3 and female = 2	50 min, 2 sessions per week for 2 months	Baseline, postintervention, and 8 weeks after the treatment	Descriptive data showed an improvement of the motor function of the upper limb items (26 ± 19.5) and total score (36.6 ± 20.2) of the scale.	Effective	The results suggest that patients had motor learning retention, achieving a sustained benefit through the technique.
51	Park JH and Park JH [65]	2016	Nintendo Wii Fit	Virtual reality game	Mobilization of the limbs	Upper extremity	RCT	30	Male = 16 and female = 14	30 min, 5 sessions per week for 4 weeks	Baseline and postintervention (after 4 weeks)	There were significant differences in the changes between the two groups in the FM (*p* < 0.05), BBT (*p* < 0.05), and MAL-QOM (*p* < 0.05). FM pre:49.3 and FM post: 54.4 (Fugl–Meyer Assessment)	Effective	Game-based virtual reality movement therapy alone may be helpful to improve functional recovery of the upper extremity, but the addition of MP produces a larger improvement.
52	Hocine N et al. [8]	2015	PRehab	Video game	Mobilization of the limbs	Upper limb	RCT	6	AgeM = 60.66: male = 4 and female = 2	20 min, for 2 weeks (3 sessions)	Baseline and postintervention	It revealed a significant effect of the difficulty strategy on patient performance (Wilks' Lambda = 0.10; *F* = 2.38; *p* < 0.02).	Partly effective	The results of the experiment show that dynamic adaptation technique increases movement amplitude during a therapeutic session.
53	Bower KJ et al. [66]	2014	Nintendo Wii Fit	Not mentioned	Balance training Mobilization of the limbs	Upper limb and lower limb	RCT	30	AgeM = 63.6: male = 17 and female = 13	45 min, 3 sessions per week over 2–4 weeks	Baseline, two weeks, and four weeks	Improvements were observed in the majority of secondary outcomes over time in both groups. The balance group participants demonstrated greater improvements in Wii balance board-derived measures with small to large effect sizes (*d* = 0.30–1.00) at four weeks (*p*=0.007 − 0.048).	Partly effective	Specific activities targeted at balance training are potentially effective for improving standing balance.
54	Brown EVD et al. [67]	2014	Peggle	Video game	Balancing training	Upper extremity	RCT	9	AgeM = 60: male = 5 and female = 4	45 min, 5 sessions per week for 4 weeks	Baseline and postintervention assessments, approximately 4 weeks apart, before system use	No differences were found across time on any of the WMFT subscales or the CAHAI-9 WMFT functional activity score: A1: 1.79 ± 0.71; A2: 1.77 ± 0.68; A3:1.79 ±0.66	No effective	This study had limited changes in kinematic and activity level outcomes
55	Slijper A et al. [68]	2014	Not mentioned	Video game	Mobilization of the limbs	Upper extremity	Before and after trial	11	AgeM = 58: male = 5 and female = 6	5 weeks, mean time: 1070 min	Baseline, during, postintervention, and follow-up16–18 weeks after the treatment phase	FMA-UE A-D (motor function) showed significant improvements in the upper extremity function between baseline (A1) and posttest (A2) (0.005) as well as a follow-up (<0.0001). Fugl–Meyer A-D: preintervention: 44, intervention: 49 , postintervention: 51	Effective	The results indicate that computer game-based training could be a promising approach to improve upper extremity function.
56	Chen CC et al. [69]	2017	Not mentioned	Virtual reality game	Muscular strengthening Mobilization of the limbs	Upper limb	Before and after trial	21	AgeM = 55.7: male = 14 and female = 7	60 min, 3 sessions per week for 8 weeks	Baseline and postintervention	The statistical results confirmed a significant effect of treatment. FMA: baseline: 30.35 ± 13.8. After intervention: 38.80 ± 14.61	Effective	Finding suggests that VR-based rehabilitation can induce significantly kinetic changes than facilitate recovery.
57	Lee MM et al. [70]	2018	Nintendo Wii Fit	Virtual reality game	Balance training Mobilization of the limbs	Upper extremity	RCT	30	AgeM = 61.56: male = 18 and female = 12	30 min, 3 sessions per week, for 5 weeks	Baseline and postintervention one day after the five-week intervention period	MFT was significantly improved in both groups compared with baseline values (*p* < 0.05). Pre: 8.93 ± 1.53; post: 11.40 ± 2.47	Effective	Game-based VR Canoe paddling training is an effective rehabilitation therapy that enhances postural balance and upper extremity function.
58	Park DS et al. [71]	2017	Microsoft Xbox 360 Kinect	Virtual reality game with Kinect	Mobilization of the limbs Balance training Motor function	Lower extremity	RCT	20	AgeM = 63.65: male = 10 and female = 10	30 min, daily sessions for a 6-week period	Baseline and postintervention	The pre-to-post difference scores on BBS, TUG, and 10 mWT for the intervention group were significantly more improved than those for the control group (*p* < 0.05).	Effective	Evidence supports the use of additional VR training with the Xbox Kinect gaming system as an effective therapeutic approach for improving motor function.
59	Park JS et al. [72]	2019	Not mentioned	Video game	Muscular strengthening Motor function	Hand	RCT	43	AgeM = 59.43: male = 26 and female = 17	30 min, 5 sessions per week, for 6 weeks	Baseline and postintervention	After training, hand strength, MFT, and BBT were improved in the experimental group compared to the control group (*P* < 0.001, both). MFT: pre: 12.91 ± 5.73; post: 16.23 ± 5.95	Effective	Game-based exercise is more effective than manual exercise in improving muscle strength, motor function, and compliance in stroke patients.
60	Ahmadi HS et al. [73]	2019	E-Link	Virtual reality game	Mobilization of the limbs	Upper limb	Nonrandomized clinical trials	30	AgeM = 55.24: male = 20 and female = 10	40 min, 3 sessions per week, for 4 weeks	Baseline and postintervention	The finding shows the improvement of upper limb motor function, tone, and range of motion in this group. Mean differences: FMA (total score); intervention: 6.53; control: 3.86	Effective	Computer games can improve upper limb motor function, muscle tone, and the range of motion in stroke patients.

FMA-UE, Fugl–Meyer Assessment for Upper Extremity; WMFT, Wolf Motor Function Test; IMI, Intrinsic Motivation Inventory; IADL, Lawton of instrumental activities of daily living; SIS, Stroke Impact Scale; B-stage, brainstorm stage; MMT, manual muscle testing; AP-axis, anterior-posterior axis; CIMT, constraint-induced movement therapy; GR, gesture recognition; NWF, Nintendo Wii Fit^TM^ game; FU, follow-up; FMA-LE, Fugl–Meyer Assessment; BESTest, Balance Evaluation Systems Test; AT, after training; 10MWT, 10-meter test of walking score; CoP, center of pressure; AP sway, sway kinematics in the anterior-posterior; BBS, the Berg Balance Scale; FABS, Fullerton Advanced Balance Scale; TUG, Timed Up and Go; FM, Fugl–Meyer; ARA, Action Research Arm; UE, upper extremity; VGG, video game group; TG, traditional group; IQR, interquartile range; FMA-UL, Fugl–Meyer upper limit assessment; OTSVR, off-the-shelf virtual reality; TTP, time-to-peak; VR, virtual reality; FR, forward reach; MAL-QOM, Motor Activity Log Quality of Movement; FMA, Fugl–Meyer Assessment; MI, Motricity Index; AROM, active range of motion; BI, Barthel Index; SG, serious games; QFG, quadriceps femoris; HSG, hamstrings; PNF, proprioceptive neuromuscular facilitation; WVRT, Wii Fit virtual reality training; GBT, general balance training; EG, experimental group; ES, effect sizes; BBT, Box and Block Test; MP, mental practice; CAHAI-9, Chedoke Arm and Hand Activity Inventory-9; MFT, manual function test; RCT, randomized controlled trial or randomized control trial.

**Table 3:** Distribution of studies based on publication type.

Journal/conference name	Conference	Journal
Clinical Rehabilitation		5
Journal of Stroke and Cerebrovascular Diseases		4
Archives of Physical Medicine and Rehabilitation		4
Games for Health Journal: Research, development, and clinical applications		4
Disability and Rehabilitation		2
Journal of NeuroEngineering and Rehabilitation		2
NeuroRehabilitation		2
IEEE Transactions on Neural Systems and Rehabilitation Engineering		2
International Journal of Environmental Research and Public Health		2
Journal of Medical and Biological Engineering		1
International Medical Journal of Experimental and Clinical Research		1
American Journal of Physical Medicine and Rehabilitation		1
Computers in Biology and Medicine		1
Journal of Central Nervous System Disease		1
BioMed Research International		1
Brain Impairment		1
European Journal of Physical and Rehabilitation Medicine		1
User Modeling and User-Adapted Interaction		1
Frontiers in Psychology		1
Iranian Rehabilitation Journal		1
Journal of Physical Therapy Science		1
Journal of Healthcare Engineering		1
Annals of Physical and Rehabilitation Medicine		1
Journal of Motor Behavior		1
American Academy of Physical Medicine and Rehabilitation		1
Journal of Patient-Centered Research and Reviews		1
Restorative Neurology and Neuroscience		1
Stroke		1
Medical Science Monitor		1
Neurorehabilitation and Neural Repair		1
Somatosensory and Motor Research		1
The Journal of Physical Therapy Science		1
International Journal of Stroke		1
Virtual Reality		1
International Journal of Neuroscience		1
In Proceedings of the 3rd 2015 Workshop on ICTs for improving Patients Rehabilitation Research Techniques	2	
Proceedings of the IEEE International Conference on Advanced Materials for Science and Engineering	1	
In 2019 International Conference on Robotics and Automation in Industry	1	
2019 Fifth International Conference on Advances in Biomedical Engineering (ICABME)	1	
International Conference on Virtual Rehabilitation	1	
2017 International Conference on Applied System Innovation (ICASI)	1	
Total	7	53

**Table 4:** Distributions of studies of publication years and country.

Row labels	Column labels								
	2013	2014	2015	2016	2017	2018	2019	2020	Total
Australia		1	1						2
Brazil^*∗*^		1	2	1		2	2	1	9
Canada		1	1				1		3
China				1					1
France			1				1		2
Iran							1		1
Israel		1	2	1					4
Italy		1						1	2
Lebanon								1	1
Malaysia							1		1
Netherlands		1		1					2
New Zealand		1							1
Pakistan							1		1
Republic of Korea^*∗*^			1	4	2	2	4		13
Spain								1	1
Sweden		1							1
Taiwan^*∗*^	1	1			1	2	1		6
Turkey			1			2			3
UK				2					2
USA		1		1		1	1		4
Grand total	1	10	9	11	3	9	13	4	60

^∗^3 countries with the highest number of study prints.

**Table 5:** Distribution of studies based on the type of study and effectiveness.

Row labels	Effectiveness
Effective	41
Before and after trial	13
Nonrandomized clinical trials	2
RCT	26
Not effective	3
RCT	3
Partly effective	16
Before and after trial	3
RCT	13
Total	60

## Data Availability

All data generated or analyzed during this study are included within this article.
